# Analysis of the Style Characteristics of National Dance Based on 3D Reconstruction

**DOI:** 10.1155/2022/2419175

**Published:** 2022-06-20

**Authors:** Dongqi Zhang

**Affiliations:** Yangtze University, Jingzhou 434020, China

## Abstract

National dance is an important symbol of national spiritual culture, as it embodies each nation's unique history, living habits, ideology, and culture. Many Chinese ethnic groups have developed their own dance forms and styles, each with their own set of charms. Strengthening our understanding of its style and characteristics is critical to our understanding of the national dance. To begin with, this paper proposes a patch-based multiview stereo reconstruction scheme that can accurately reconstruct 3D character models. The movement capture system then collects national dance movement data and uses them to drive a three-dimensional character model that generates dance visual animation. In the human skeleton model, a spatial-temporal HMM (hidden Markov model) is proposed that not only studies the temporal information of human movements but also the spatial information of adjacent connection points. The recognition rate of this algorithm increases to 95.68 percent when the number of setting points is increased to ten and to 98.28 percent when the number of setting points is increased to twenty, according to the research. The experimental results show that the 3D reconstruction model of ethnic dance developed in this paper is capable of meeting the goal of ethnic dance digitalization while being simple to use, being low in cost, and with a good display effect.

## 1. Introduction

Three factors make up the essence of dance style: formal characteristics, thoughts, and images of dance works. They are concerned not only with the expression of the external form of dance works but also with the transmission of spiritual ideas. Many factors influence the formation and development of a dance style, including the social environment, history, and culture, as well as the personal preferences and aesthetics of the dancers. The styles and characteristics of different national dances are obviously different, influenced by regional, national psychology, culture, and other factors. People will gain a better understanding of ethnic dance style characteristics by comparing the style characteristics of different ethnic dances. National dancers use special costumes or auxiliary props such as a stage to assist dancers in performing and silk to express dance images, in addition to using body movements to express national dance culture. The effective arrangement of dance movements and efforts to use the arrangement and flexible design of shapes to form a good dance performance image share many similarities with national dance art and painting art. The lines produce products that satisfy the aesthetics, interesting dance steps, and emotional resonance of the audience.

National dance has a long and ancient history as a phenomenon of dance culture and embodies a specific style and a specific form, as well as historical changes and the development of the times in a specific period, i.e., the development of the times has a far-reaching impact on the national dance culture. To demonstrate the national dance, Piniés et al. used 3D modeling and human motion capture technology, and the model used in the dance was an animation model drawn by hand [1]. Ma et al. proposed a dance training system that combines motion capture and virtual reality by capturing imitation motion, projecting it on the screen using virtual reality technology, and providing feedback, but there occurred a large error in capturing motion [2]. Jones et al. proposed to perform three-dimensional convolution in the CNN (Convolutional Neural Network) convolution layer, in order to capture the distinguishing features of spatial and temporal dimensions [3]. By extracting 16 joint points, Liu et al. were able to perform motion tracking and attitude analysis. Because the human body's movements are flexible, simply changing the joints will result in a large error in recognizing the movements of the human body [4]. Werner et al. used the metric learning algorithm twice during the time-consuming model training stage. This means that achieving the real-time recognition effect for an unfamiliar action is difficult for the algorithm [5]. Furthermore, because this type of algorithm must make complex decisions in order to eliminate a large number of false 3D graphics primitives, the search volume is too large and the efficiency is too low, making it unsuitable for widespread use. It is the most effective means of improving the efficiency of the bottom-up recognition algorithm by aligning it with engineers' drawing methods and starting from a higher level of graphic semantics.

Video technology research has become one of the hottest topics in academia in recent years. Video motion recognition is one of the most important video technologies for the application of video intelligence, and it is widely used in many fields [6, 7]. As a result, using 3D reconstruction technology to protect Chinese national dance art and culture is critical. The national dance artists are reconstructed using 3D reconstruction technology [8], their images are saved in digital form on the computer, and a model of national dance artists driven by dance scores is imported. The underlying data are selected and analyzed in the feature extraction stage, and the action information is modeled on the data to obtain the human action pattern. It is a crucial component of human motion recognition that has a direct impact on the accuracy and robustness of the system. It investigates not only the time series data of human movement but also the spatial data of adjacent connection points in the human skeleton model, in order to better reflect the fundamental law of feature distribution.

### 1.1. Main Research Contributions

1. This document combines camera image array and Kinect principle to collect depth images and calculates the 3D point cloud coordinates and normal vectors of depth images. Then, this paper uses the camera pose matrix estimation method with edge feature points as the auxiliary relationship to realize point cloud matching, and the generated point cloud is triangulated to form a triangular surface model.
2. People should not only judge the type of action according to the image when the action is still but also pay attention to the whole changing process of the action from the beginning to the end. In this paper, a human motion recognition algorithm based on 3D joint space-time information is proposed. The algorithm extends the one-dimensional hidden Markov model, which studies time series information, to spatial time series HMM, which not only studies the time series information of actions but also studies the spatial information of events.

### 1.2. Structural Arrangement

Section 1 introduces the research background and significance and then gives the main work of this paper. Section 2 mainly introduces the related technologies of 3D reconstruction. Section 3 puts forward the concrete methods and implementation of this research. Section 4 verifies the superiority and feasibility of this research model. Section 5 is the summary of the full text.

## 2. Related Work

### 2.1. Research on 3D Reconstruction Technology

3D reconstruction is an important part of the field of artificial vision, in which the recovery of 3D structures of objects and scenes from 2D image sequences based on motion information has always been an important research content of 3D reconstruction. In order to get more detailed information from the model, it is necessary to reconstruct a dense point cloud. Therefore, it is very important to solve the problem of dense pixel matching in image sequences.

Ma et al. proposed an energy function, which contains not only a constant brightness term but also a regularization term, which can supplement the optical flow information of weak texture areas [9]. Hernando et al. adopted effective duality based on optimization scheme and extended it to video registration of multiframe optical streams by establishing a long-term temporal coherence model with subspace constraints [10]. Han et al. proposed that the subspace constraint should be regarded as an implicit long-term trajectory regularization term in the whole video, and the time-consistent optical flow can be obtained [11]. Lu et al. proposed using subspace constraints to build a multiframe optical flow model and made a clear reasoning on occlusion [12]. However, this method is limited by the hard subspace constraint of the known principal component analysis base, which is calculated by sparse feature tracking.

The method of model reconstruction through the software can provide abundant components and functions by the software itself, and it is convenient to construct the Wang Wei model, which provides convenience for the design of the article model. Kottkamp et al. proposed an automatic surface generation system [13]. The system uses a handheld camera to collect image sequences, and through multiview feature matching, it can automatically complete camera calibration and layered reconstruction of object surface. Boden et al. constructed the RGB-D mapping system by using the depth and color information collected by Kinect [14]. The system combines battery correction and visual feature matching and realizes the postregistration of three-dimensional point clouds. Then, through closed-loop detection and global optimization, the indoor scene can be reconstructed in real time. Chen et al. realized real-time 3D reconstruction by using mobile Kinect and studied the physical interaction and multitouch of the reconstructed scene [15].

### 2.2. Research on Human Motion Recognition Technology

The features of human motion recognition learned by traditional methods cannot cope with the troubles caused by complex scenes, and the problems to be solved are limited. The way of deep learning conforms to the mechanism of human perception of the world. When there are enough samples, the features learned through deep network often have certain semantic features.

Yin et al. divided the human skeleton into five parts, represented by five subnetworks, and then fused them at the high level. An end-to-end recurrent neural network method based on the skeleton is proposed for human body recognition [16]. Iosifidis et al. put forward a new cyclic attention neural network, which uses separated spatial attention to improve the accuracy in the data set [17]. Almazán et al. put forward a dance training method based on systematic desensitization, defined the function of systematic desensitization training, and concluded that this method can help athletes to master sports dance skills [18]. Wang applied support vector machine to motion recognition, and they classified the extracted local feature vectors linearly. Later, many researchers used support vector machine in the recognition process [19]. Wang et al. combined the features of skeleton and contour, considered the boundary of contour itself, and used the background removal method to obtain contour [20]. Then, the histogram of human body shape is calculated by a radial algorithm centered on silhouette, and the final descriptor is obtained by combining the two features. Chang et al. used inertial sensors and depth cameras to capture the actions of cooking food (such as cutting food, subpackaging food, and eating food) [21]. Referring to the acceleration measured with the wearable inertial sensor, the coordinates and displacements of the human wrist, elbow, and shoulder can be estimated according to the depth data.

## 3. Methodology

### 3.1. Three-Dimensional Reconstruction of the National Dance Style Characteristics

#### 3.1.1. Overall Framework

The primary goal of the national dance deductive process is to use the image deductive process to allow the audience to truly experience and feel the allure of dance as an art form. Each nation's physical formation and dynamic characteristics are not only closely related to the nation's historical development but also the result of artistic creation. Dance is thus not only an artistic expression but also a symbol of traditional culture and customs. Every feature of each historical stage is reflected in national dance, which has always been the carrier of popular culture. In a unique way, it preserves and accumulates cultural factors at various historical stages. The model's accuracy is always inversely proportional to the amount of data stored. A portion of the storage space will be sacrificed in order to achieve high accuracy, and the compression of the storage space will inevitably result in a decrease in accuracy. As a result of the discrepancy between the amount of data and the model's accuracy, the strain reference template is chosen for the measured point cloud. The first box's point cloud template is arbitrary and can be a standard template. The previous frame's point cloud is used as the reference template for the next frame after nonrigid body registration, and then, the rigid body's point cloud registration method with two viewpoints is used for preregistration. This is to strike a balance between accuracy and data volume so that the final model can satisfy both computers and users.

Using the depth data collected by mobile Kinect, high-quality 3D models can be reconstructed in real time. The technical framework of the Kinect Fusion system is shown in Figure 1.

Firstly, the system collects the original depth data through Kinect and then calculates the unit coordinates and normal vectors from the spatial point cloud. Then, the absolute camera pose is calculated by iterative algorithm, and the point cloud registration operation is carried out. In the process of point cloud merging, different from the previous simple point cloud merging methods, the system uses truncated symbolic distance function to map the point cloud data into a global cube to realize the merging. Finally, the ray tracing method is used to model the surface according to the current camera pose.

Because the obtained depth map contains some holes, it is necessary to repair the depth map in order to improve the quality of subsequent reconstruction. In this paper, the method of joint bilateral filtering is used to draw depth data. Its basic idea is to use the RGB image as the guide map and fill the missing information in the depth map with its full-edge information.

The filtered depth map is expressed as

(1) $$\begin{array}{c} D_{x}^{\prime }=\frac{\sum_{ij}w_{i,j}^{s}w_{i,j}^{c}w_{i,j}^{z}}{\sum_{ij}w_{i,j}}, \end{array}$$

where *w*_*i*,*j*_^*s*^,  *w*_*i*,*j*_^*c*^,  and  *w*_*i*,*j*_^*z*^ is the spatial weight, color weight, and depth weight, respectively.

The data processing flow of the system mainly includes three parts: calibration, acquisition, and registration, as shown in Figure 2.

After the system is started, first initialize the system parameters, setting the Kinect depth frame resolution to 650 × 460 and the frame rate to 20 frames per second, and initialize Kinect Fusion-related parameters. In the acquisition stage, Kinect Fusion integrates them into their global surface model system and uses the ICP (Iterative Closest Point) algorithm.

Estimation of the current position of Kinect: in the registration stage, two point clouds are fitted to the same coordinate system, which provides a good starting position for the subsequent ICP algorithm and improves the registration accuracy. In the calibration stage, the point clouds obtained by two Kinect cameras are adjusted to the same coordinate system. The calibration process only needs to be done once after the hardware platform of the system is built.

#### 3.1.2. Point Cloud Registration

Point cloud registration is the key link of network reconfiguration technology, and the accuracy of point cloud registration directly affects the quality of the reconfiguration model. Because the accuracy of image processing is usually high, this step needs a lot of calculations, so the execution efficiency becomes one of the criteria to judge the algorithm. Besides efficiency, the accuracy and completeness of reconstruction must also be considered, because these factors determine the quality of the point cloud. In the process of recording consecutive frames, the body shape parameters of the same measured object must be the same. Firstly, the shape parameters of the standard model are selected as reference elements and then optimized according to the cost function, which is optimized frame by frame.

PMVS (Patch-Based Mufti View Stereo) algorithm is the best multiview stereo reconstruction algorithm at present. In addition, in order to distinguish between rendering and sparse reconstruction, this step is also called dense reconstruction. PMVS only reconstructs rigid structures. It will automatically ignore nonrigid structures, such as pedestrians in front of buildings. Given a set of oriented 3D points, the 3D coordinates and normal of each point are estimated. When the Kinect acquisition scene is mainly composed of walls and other planes, the ICP algorithm adopted by Kinect Fusion will terminate the iteration problem ahead of time, and the camera pose cannot be accurately estimated at this time, which will affect the results. It is not difficult to imagine that this problem can be solved by adding other corresponding nearest point pair selection methods. Therefore, this paper adopts the method of adding the edge features corresponding to the nearest points to avoid this problem.

Because the number of edge feature points in the registration process is much smaller than the number of nearest points corresponding to the original method, the error function between the nearest points of the edge is relatively weak. Here, the weight coefficient *α* is used to amplify the edge characteristic error function and increase its proportion in the total error function. So the final error function is shown in the following equation:

(2) $$\begin{array}{c} E{\;}^{\prime }\left(T_{g,i}\right)=E_{1}+\alpha E_{2}, \end{array}$$

where it is the error function before modification, namely,

(3) $$\begin{array}{c} E_{1}={\sum_{u}\left\|{\left(T_{g,i}{\dot{V}}_{i}\left(u\right)-{\hat{V}}_{i-1}^{g}\left(\hat{u}\right)\right)}^{T}\cdot N_{i-1}^{g}\left(\hat{u}\right)\right\|}_{2},\\ E_{2}=\sum_{q}{\left\|T_{g,i}{\dot{V}}_{i}\left(q\right)-{\hat{V}}_{i-1}^{g}\left(\hat{q}\right)\right\|}_{2}. \end{array}$$

From the operations given above, we can get the final error function *E* ′(*T*_*g*,*i*_), which is consistent with the original error function of Kinect Fusion, and *E* ′(*T*_*g*,*i*_) can also be transformed into linear equations for least square optimization.

The center coordinate and normal vector of the patch are optimized to maximize the average correlation coefficient. In the optimization process, the center point of the patch is fixed on the ray of the reference image and the optimization degree of freedom is 3. The *z* coordinate of the center of the patch represents the two angles *α* and *β* of the normal vector. The equation of the slope is shown as follows:

(4) $$\begin{array}{c} a\left(X-X_{c}\right)+b\left(Y-Y_{c}\right)+c\left(Z-Z_{c}\right)=0. \end{array}$$

The relationship between normal and direction angle is *a*=cos*α*cos*β*, *b*=sin*α*cos*β*,  and *c*=sin*β*.

#### 3.1.3. Body Shape and Posture Estimation

The Poisson reconstruction method is used to reconstruct the surface of the recorded point cloud. Poisson reconstruction can consider all sampling points globally and has good robustness. After the surface is reconstructed, texture mapping is performed according to the vertices of the human mesh and the nearest neighbors of the human point cloud. For the vertex of each patch in the model, we find the nearest point in the point cloud, calculate the distance between the corresponding points, and assign the texture coordinates of that point to the vertex if it is less than the threshold. Considering the extensive research value and application prospect of the 3D human body model, this section proposes a method of human body model reconstruction combined with the human body model for nonrigid reconstruction of the dynamic human body. SMPL (Skinned Multiperson Linear) can accurately represent various postures and body shapes of the human body according to the deformation of skin apex, can simulate the bulge and depression of human muscles and other tissues during limb movement, so as to avoid surface deformation during movement, and can accurately describe the human body. Stretched and contracted muscles show the same soft tissue movement as real people.

Through rigid body registration, the two models are preregistered, and then the shape and posture parameters of SMPL are optimized to obtain the final model. The cost parameters are constructed as follows:

(5) $$\begin{array}{c} E\left(\beta ,\theta \right)=\lambda_{m2s}E_{m2s}+\lambda_{\beta }E_{\beta }\left(\beta \right)+\lambda_{\theta }E_{\theta }\left(\theta \right). \end{array}$$

Among them, *E*_*β*_ in the cost function is the prior constraint term of body shape and *E*_*θ*_ in the cost function is the constraint of posture, which helps to prevent unnatural posture. The obtained body shape parameters and posture parameters are input into the SMPL generation model, and a complete three-dimensional human body model is obtained.

The constraint term *E*_*m*2*s*_ represents the sum of the distances of the corresponding points between the reconstructed points and the standard model:

(6) $$\begin{array}{c} E_{m2s}\left(M,P\right)=\sum_{m_{i}\in vis\left(M\right)}\rho \left(\min\left\|m_{i},v\right\|\right). \end{array}$$

Here, *M* is the model surface, *P* is the scanning point cloud, function *vis*(*M*) represents the effective visible model vertex, *m*_*i*_ is the effective point on *P*, *ρ* is the robust Geman–McClure function, and *v* is the point corresponding to *m*_*i*_ point on the SMPL model. *λ*_*m*2*s*_ is its weight term.

### 3.2. Dance Movement Recognition

#### 3.2.1. Feature Extraction

National dance is a form of time and space coexistence art. It, like other straight tree arts, has cultural and individual characteristics that are connected through communication. The passage of time and space has brought about significant changes in people's lives and cultures. National dance should be based on current events. At the same time, folk dance follows the rhythm of the times and incorporates its characteristics. The theme and dance form were innovated and arranged in accordance with China's different revolutionary histories and modern opening periods, reflecting the characteristics of the times at the time. The goal of extracting local features in human motion recognition is to pique people's curiosity. In the part of a motion that changes significantly, there is no need to locate and track the entire human body. External environmental factors such as the change in human body shape, the change in shooting angle, the change in illumination, and the problem of occlusion have strong anti-interference properties.

In the experiment of this chapter, (*x*_*i*_, *y*_*i*_, *z*_*i*_) is used to represent the three-dimensional coordinate of the *i*th bone joint and *J*=[*J*_1_, *J*_2_,…, *J*_*M*_] represents the selected *M* bone joints. The calculation method of displacement vector features is as follows:

(7) $$\begin{array}{c} d_{i}^{t}=\frac{J_{i}^{t+1}-J_{i}^{t-1}}{\Delta T},\;t=1,2,\ldots ,N,\;i=1,2,\ldots ,M, \end{array}$$

where*J*_*i*_^*t*^ represents the coordinate of the *i*th bone joint in the *t* frame, *N* represents the serial number of the frame in which the bone joint is located, and *M* represents the corresponding label of the selected bone joint. Δ*T* represents the time interval between the *t*+1 frame and the *t* − 1 frame.

Content-based retrieval technology has been proved to be very effective and fast in similarity search of large-scale data. Therefore, this section is devoted to extending the retrieval technology to real-time motion recognition. General templates representing various categories can be used as template patterns to directly match and identify test actions.

Assume that *x* and *y* represent a frame of the test sample and the general template, respectively, to support the similarity calculation:

(8) $$\begin{array}{c} h_{p}\left(x,y\right)=\left\{\begin{array}{cc} 1, & x_{p}\in y_{p},\\ 0, & \text{otherwise.} \end{array}\right. \end{array}$$

Here, if the two *x* and *y* do not match, *s*(*x*, *y*) is no longer assigned to zero, but a negative value, and *h*_*p*_(*x*, *y*) − 5 is given as punishment, thus enhancing the difference between different actions.

In the process of recognition, each part of it is searched in its corresponding key table in turn. The accumulated scores of these results can be used as the identification basis, and the specific identification process is shown in Figure 3.

After the previous steps, the key frame is represented by a five-dimensional vector, where each dimension represents the pose mapping of a part of the frame. For each dimension, we look for its match on its corresponding key. Therefore, five sets of search results are returned for these five dimensions. Therefore, we need to further analyze these search results and find the matching results from the intermediate frames. The input frame can always find as many matches as possible, which leads to the accurate classification of similar actions. Finally, input action recognition is determined by the general template with the highest performance score.

#### 3.2.2. Action Classifier Design

HMM (hidden Markov model) is a dynamic model based on stochastic process and probabilistic observation. It is widely used in the recognition of various dynamic process systems involving state transition, such as speech recognition, handwriting recognition, and motion recognition. Its basic assumptions include the output independence hypothesis and the Markov hypothesis. The value is implicit, and it is one of some finite sequence of states. Markov hypothesis means that the current state completely depends on the state of the previous moment, and there is a fixed probability of this dependence between states.

Evaluation is the first problem to be solved in the motion recognition algorithm based on HMM, because given the observation sequence *O* and multiple HMMs, it is necessary to judge which HMM produced the observation sequence *O* according to the evaluation results.

There are two solutions to the evaluation problem: the forward algorithm and the backward algorithm. The Markov hypothesis is extended to the two-dimensional case. The state of the feature block depends on the state of the left feature block and the state of the upper feature block. There is a fixed probability between these states.

Both forward probability and backward probability can be calculated effectively by recursion. Unlike the new forward algorithm proposed in this paper, the iterative sequence of backward algorithm is from right to left and from bottom to top. The backward algorithm iteratively calculates *ϕ*_*i*_^*w*+1^(*m*, *x*) and *β*_*i*+1_^*w*^(*m*, *n*), which represents the backward probability of the joint state of adjacent feature blocks. Their definitions are as follows:

(9) $$\begin{array}{c} \beta_{i+1}^{w}\left(m,n\right)=p\left(o_{i+1}^{w+1,\ldots ,W},O_{t+2},\ldots ,O_{T}|q_{i}^{w}=s_{m},q_{i+1}^{w}=s_{n}\right),\\ \phi_{i}^{w+1}\left(m,x\right)=p\left(O_{i+1},\ldots ,O_{T}|q_{i}^{w}=s_{m},q_{i}^{w}=s_{x}\right). \end{array}$$

## 4. Experiment and Results

In order to quantitatively compare the 3D SMPL human body models reconstructed by this method, this section uses the shadow recovery shape 3D reconstruction method to establish the standard 3D human body template and adds additional illumination constraints on the basis of this method. In order to optimize the depth value, this method integrates the illumination information of the object surface and the generated 3D model is smoother and contains more detailed information of the object surface.

Then, the three-dimensional human body model reconstructed by the first two methods is registered with the standard template, and the nearest geometric distance between the reconstructed model point and the standard template is calculated and represented by pseudo-color. By comparing the root mean square values of the generated model and template, the similarity between the model and template can be effectively reflected. The error comparison of the former two methods is shown in Figure 4.

According to the calculation of Figure 4, the average root mean square error of this method is 2.23 times that of this method and the reconstruction effect of this method is better.

For each group of data sets, we conduct a user-independent group action pattern recognition experiment, and we select three collected samples as training sets and the other two as test samples. As shown in Figures 5 and 6, for each action type, only the first two training samples are selected for each captured topic for training; that is, there are only 6 training samples for each action type.

It can be seen from the results that the recognition accuracy of this method is the highest among all methods. As far as human perception is concerned, they belong to the same action category, but due to different arm actions, the action data values may be quite different. Therefore, when these actions are calculated and recognized as a whole, the recognition accuracy will be seriously affected and our limb-based segmentation method can avoid this shortcoming.

In this section, on the basis of the above experiments, some extended experiments are made.  Table 1 gives the comparison of the algorithm proposed in this paper and the training time of a single sample in each stage of reference [19–21].

It can be seen from Table 1 that the average training time of the model in [19] for a single sample is more than 20 times higher than that of the algorithm in this paper. The amount of data in this database is relatively small, so this time cannot be ignored for a database with a relatively large amount of data. It can be concluded that the algorithm in this paper can basically recognize human movements in real time. More importantly, the algorithm in this document does not need human intervention. According to different databases, the parameter values can be automatically adjusted according to the input data, and the adaptability is strong.

In order to reduce the randomness of the clustering process, nine people are used for training and one person is used for testing in the database, which is a one-time cross-validation method.  Table 2 shows comparison with the other literature studies.

As can be seen from Table 2, the recognition rate of this algorithm basically exceeds that of all the current literature. It is easy for an algorithm to achieve a high recognition rate in the database, but it is very difficult to increase it by a few percentage points on the existing basis.

The auxiliary training method collects the coordinate points of each trainer's motion joints and compares them with the standard movements. The Kinect is used to collect the position of the trainer's motion coordinates, and the error values of the motion joint coordinates obtained by the three methods are compared to assist the dance method. Compared with the data collected by Kinect, the detailed analysis of joint angle capture in motion capture shows the experimental results in Figure 7.

In Figure 7, the method designed in this paper is more accurate in angle capture than other comparison methods. It can be known that the analysis method of folk dance style characteristics based on 3D reconstruction designed in this paper has higher accuracy in capturing the trainer's movement position and can form a more accurate contrast with the standard movement, thus realizing error correction in auxiliary training.

The experiment will investigate the influence of test sample noise on spatio-temporal HMM recognition performance. The test sample feature space is composed of Gaussian noise with different signal-to-noise ratios. At this time, the number of training samples is set to 50% of the total number of samples. In the experiment, feature information from different joint points is used to represent the features of the human body model and the influence of feature dimensions on the recognition rate of the model is tested. The results are shown in Figure 8.

The change of curve reflects the influence of the dimension change of skeleton model features on the recognition algorithm. The larger the dimension, the richer the skeleton model features. When the feature dimension increases, the recognition rate increases, while the recognition rate of one-dimensional Markov model algorithm decreases. When the number of joints increases to 10, the recognition rate of our algorithm increases to 95.68%, and when the number of joints increases to 20, the recognition rate of our algorithm increases to 98% and 28%. When the feature dimension is small, the reason for the low recognition rate of our algorithm in this paper is that the spatial dependency between low-dimensional feature blocks is fuzzy and the dependency is easily affected by noise in the training feature space, which will affect the performance of our algorithm. Experimental results show that the proposed algorithm is superior to the one-dimensional Markov model algorithm in recognition rate and robustness in solving high-dimensional human motion recognition problems.

## 5. Conclusions

Ethnic dance is a powerful reflection of a country's culture, national identity, and historical tradition. Dances of various nationalities have their own distinct styles as an important cultural card of a nation. It is necessary to understand the style characteristics of national dance in order to better understand its performance characteristics and improve its performance effect. This is done by first understanding its basic characteristics. The upper and lower parts of the human body are scanned with two Kinect depth cameras, and the two 3D point clouds obtained by scanning are spliced to create a complete 3D model of the human body. The one-dimensional hidden Markov model is extended to the spatial time series HMM in order to solve the dimension disaster caused by the three-dimensional representation of the human body. The recognition rate of this algorithm increases to 95.68 percent when the number of joints is increased to ten and to 98.28 percent when the number of joints is increased to twenty, according to the experimental results. This method is quick and simple to use, and it can be applied to augmented reality, ethnic dance style analysis, and other applications.

## Figures and Tables

**Figure 1:** System framework.

**Figure 2:** Data processing flow.

**Figure 3:** Real-time motion recognition process.

**Figure 4:** Error comparison of algorithms.

**Figure 5:** Recognition accuracy (data set 1).

**Figure 6:** Recognition accuracy (data set 2).

**Figure 7:** Comparison of joint angle values of trainers.

**Figure 8:** Influence of feature information of different number of joints on recognition rate of different algorithms.

**Table 1:** Training time comparison.

Method	Feature extraction (ms)	Feature processing (ms)	Training classifier (ms)
Methods of this paper	6.693	0.524	6.632
Literature [19]	6.358	6.012	2012.214
Literature [20]	10.332	18.324	1869.367
Literature [21]	7.213	9.668	2231.47

**Table 2:** Comparison between identification results and mainstream methods.

Method	Recognition rate (%)
Methods of this paper	88.6
Literature [19]	93.2
Literature [20]	90.7
Literature [21]	97.8

## Data Availability

The data used to support the findings of this study are available from the author upon request.
